# Real-World Efficacy and Safety of Sintilimab-Based Regimens against Advanced Esophageal Cancer: A Single-Center Retrospective Observational Study

**DOI:** 10.1155/2022/7331687

**Published:** 2022-08-05

**Authors:** Chenyu Wang, Linzhi Jin, Xinyu Cheng, Runchuan Ren, Anping Zheng, Anlin Hao, Nengchao Wang, Jinwen Zhang, Fuyou Zhou, Yaowen Zhang

**Affiliations:** Department of Radiotherapy, Anyang Tumor Hospital, The Affiliated Anyang Tumor Hospital of Henan University of Science and Technology, Henan Medical Key Laboratory of Precise Prevention and Treatment of Esophageal Cancer, Anyang 455000, China

## Abstract

This study is aimed at assessing the sintilimab-based regimens' safety and efficacy for advanced esophageal cancer (EC) treatment in the real world. Cases of advanced EC treated with sintilimab-based regimens in the Anyang Tumor Hospital between 1 January 2020 and 1 August 2021 were retrospectively examined. Progression-free survival (PFS), overall survival (OS), disease control rate (DCR), objective response rate (ORR), and adverse events (AEs) were evaluated. Among the 50 included patients, the median PFS was 11.3 months (95% CI: 5.0-17.6 months), and the 1-year PFS rate was 49.2%. The median OS was not reached, and the 1-year OS rate was 67.1%. Complete response (CR), partial response (PR), stable disease (SD), and progressive disease (PD) were seen in 14% (*n* = 7), 46% (*n* = 23), 32% (*n* = 16), and 8% (*n* = 4) of the 50 patients, respectively. Therefore, the ORR and DCR were 60% (30/50) and 92% (46/50), respectively. The CR rate of patients with radiotherapy was higher than that without radiotherapy (25% vs. 3.8%, *P* = 0.031). The 1-year OS rate was higher in patients with radiotherapy than in patients without radiotherapy (85.9% vs. 53.2%, *P* = 0.020). The most observed AEs included anemia, decrease in white blood cell count, nausea/vomiting, and hypoproteinemia. Sintilimab-based regimens achieved good disease control and tolerance for treating advanced EC in the real world. Combined radiotherapy can improve the efficacy and deserves further study.

## 1. Introduction

The death rate of esophageal cancer (EC) ranks sixth among all malignant tumors worldwide [1]. The two main pathological subtypes of EC are esophageal adenocarcinoma and esophageal squamous cell carcinoma (ESCC), and ESCC is more than 90% in China [2]. Nearly half of EC patients are initially diagnosed at an inoperable advanced stage [3]. Systemic chemotherapy plays a vital role in the treatment of advanced patients, whose median survival time is less than one year [4]. At present, the targeted drugs used in the treatment of EC are only targeted at HER2 or vascular endothelial growth factor [5–7]. The therapeutic impact of conventional treatment plus targeted medications is still not ideal. Thus, patients with advanced EC urgently need novel and more effective treatments.

Immune checkpoint inhibitor therapy targeting programmed cell death protein 1 (PD-1) or programmed cell death ligand 1 (PD-L1) is a novel tumor immunotherapy approach that can reverse tumor immune escape [8]. Recently, immunotherapy has demonstrated great efficacy in treating non-small-cell lung cancer (NSCLC), head and neck tumors, and malignant melanoma [9, 10]. The KEYNOTE-028 and KEYNOTE-180 studies were the first to demonstrate the efficacy and safety of pembrolizumab in the treatment of advanced EC [11, 12]. Since then, KEYNOTE-181 has established pembrolizumab as an effective treatment for EC in its advanced stages [13]. Currently, several clinical trials have demonstrated the safety and efficacy of immunotherapy combined with chemotherapy or immunotherapy alone as first- or later-line treatment of advanced EC [14–17].

Sintilimab, a fully recombinant human IgG4 anti-PD-1 monoclonal antibody, is approved in China for the treatment of classic Hodgkin's lymphoma, NSCLC, and hepatocellular carcinoma [18–21]. Sintilimab is often used to treat advanced EC because of its lower cost in the real world. In this study, we assessed the efficacy and safety of sintilimab-based regimens in patients with advanced EC.

## 2. Methods

### 2.1. Patients

The study population targeted advanced EC patients who started sintilimab treatment between 1 January 2020 and 1 August 2021 in Anyang Cancer Hospital. Inclusion criteria were (1) EC confirmed by pathology, (2) recurrent or metastatic advanced EC, (3) treated with sintilimab alone or combined with other regimens, and (4) had at least one lesion that can be measured according to Response Evaluation Criteria in Solid Tumors (RECIST 1.1) [22]. Exclusion criteria were (1) suffering from second primary cancer, (2) history of autoimmune diseases, (3) uncontrolled cardiac clinical symptoms or diseases, (4) interstitial pneumonia, and (5) active hepatitis. Clinical staging was performed using the eighth edition of the TNM staging system of the American Joint Committee on Cancer (AJCC). This study was performed according to the principles of the Declaration of Helsinki and approved by the Ethics Committee of Anyang Tumor Hospital. Informed consent was not required owing the study's retrospective nature.

### 2.2. Data Collection and Outcome Assessment

Patient demographics and clinical background, blood biochemical data, treatment pattern, the efficacy of sintilimab (tumor response, progression free survival (PFS), overall survival (OS)), and the safety of sintilimab (treatment-related adverse events (AEs)) were retrospectively collected from each patient's medical records. According to RECIST 1.1, the relevant researchers assessed the tumor response. Efficacy was evaluated as complete response (CR), partial response (PR), stable disease (SD), or progressive disease (PD). Objective response rate (ORR) and disease control rate (DCR) were defined as the proportion of patients who achieved CR or PR and CR, PR, or SD, respectively. All AE severity was graded according to Common Terminology Criteria for Adverse Events (CTCAE) version 5.0 of the US National Cancer Institute.

### 2.3. Follow-Up

Follow-up began after receiving sintilimab treatment, through outpatient and inpatient system or telephone regular follow-up to understand the patient's condition. The last follow-up date was 13 April 2022.

### 2.4. Statistical Analysis

Constituent ratios were calculated to express counting data, and chi-square test was used for comparison between groups. Using the Kaplan–Meier approach, the median and estimated 95% confidence intervals (CI) for PFS and OS were computed. The log-rank test was employed to compare the survival functions of the two subgroups. *P* < 0.05 was used to determine statistical significance. All information was entered into the database and analyzed using SPSS 26.0.

## 3. Results

### 3.1. Patient Characteristics

This study comprised 50 participants, and their demographics and clinical backgrounds are detailed in Table 1. 34 (68%) of the 50 cases were males. The median age was 69 years, with a range of 41 to 85 years. Regarding histological types, the proportion of squamous cell carcinoma was 96% (*n* = 48) and adenocarcinoma was 4% (*n* = 2), respectively. Patients with metastases accounted for 72% (*n* = 36), and nonregional lymph nodes were the most common site of metastasis (42%, *n* = 21). 56% (n = 28) of patients had a history of esophagectomy, whereas 10% (*n* = 5) had a history of radiotherapy. The ECOG PS score of all patients was less than 2, of which 0 was 42% (*n* = 21).

### 3.2. Treatment Patterns

The patterns of sintilimab administration are presented in Table 2. 72% (*n* = 36) of patients received sintilimab as first-line treatment, whereas 18% (*n* = 9) received as second-line treatment. Systemic treatment models included sintilimab alone (2%, *n* = 1), sintilimab plus chemotherapy (88%, *n* = 44), and sintilimab plus antiangiogenic therapy (10%, *n* = 5). The main chemotherapeutic drugs were paclitaxel, albumin-bound paclitaxel, platinum, S-1 (tegafur-gimeracil-oteracil potassium), and irinotecan. Antiangiogenic drugs included anlotinib and apatinib. For local treatment, 48% (*n* = 24) of patients were combined with intensity modulated radiotherapy (IMRT). The median cycle and median duration of sintilimab treatment were 5 times (range: 2–27 times) and 119 days (range: 42–636 days), respectively.

### 3.3. Best Overall Respones

Figure 1(a) depicts the best changes from baseline in detectable target lesions in the 50 patients.  Figure 1(b) depicts longitudinal changes in detectable target lesions. Among the 50 patients in this study, CR, PR, SD, and PD were seen in 14% (*n* = 7), 46% (*n* = 23), 32% (*n* = 16), and 8% (*n* = 4), respectively. Therefore, the ORR and DCR were 60% (30/50) and 92% (46/50), respectively. We also examined the impact of radiotherapy on the efficacy of sintilimab. There was no significant difference in ORR and DCR between with radiotherapy and nonradiotherapy (58.3% (14/24) vs. 61.5% (16/26), *P* = 0.817; 91.7% (22/24) vs. 92.3% (24/26), *P* = 0.933), but the CR rate with radiotherapy was higher than that nonradiotherapy (25% vs. 3.8%, *P* = 0.031) (Table 3).

### 3.4. Treatment Outcomes

Figure 2 displays the Kaplan–Meier curves for PFS and OS. The median PFS for all patients was 11.3 months (95% CI: 5.0-17.6 months), and the 1-year PFS rate was 49.2%. The median OS was not reached, and the 1-year OS rate was 67.1% (Figures 2(a) and 2(b)). In this study, radiotherapy patients did not achieve the median PFS and OS. Patients without radiotherapy had a median PFS of 10.4 months (95% CI: 5.1-15.7 months), while the median OS was not reached. There was no significant difference in 1-year PFS rate between patients with or without radiotherapy (58.5% vs. 43.0%, *P* = 0.479). However, the 1-year OS rate in patients with radiotherapy was significantly higher than that without radiotherapy (85.9% vs. 53.2%, *P* = 0.020) (Figures 2(c) and 2(d)). Take a typical patient as an example. Figures 3(a)–3(j) show the outcome of sintilimab-based regimens in a patient who was initially diagnosed with advanced esophageal cancer with lung and liver metastasis. Reexamination showed that all lesions disappeared after 2 cycles of sintilimab plus albumin-bound paclitaxel, nedaplatin, and palliative radiotherapy for esophageal tumors, and positron emission tomography demonstrated the absence of tumor metabolic activity following treatment.

### 3.5. Treatment-Related Adverse Events

Three patients discontinued sintilimab due to elevated transaminases, and four patients were diagnosed with immune-mediated lung disease. No deaths attributable to treatment were observed. Of the 24 patients who received radiotherapy, 14 patients had grades 1-2 esophagitis, 1 patient had a nasogastric tube implantation due to severe swallowing pain, and none had fistula. According to CTCAE5.0, the treatment-related AEs are shown in Table 4. Most adverse events were mild (grades 1-2) and manageable. The most common grade 1-2 AEs were anemia (70%, 35/50), decrease in white blood cell count (62%, 31/50), nausea/vomiting (52%, 26/50), hypoproteinemia (42%, 21/50), decrease in neutrophil count (36%, 18/50), and pneumonia (34%, 17/50). The most common treatment − related ≥ grade 3 AEs included decrease in neutrophil count (14%, 7/50), pneumonia (10%, 5/50), and increase in alanine aminotransferase (6%, 3/50).

## 4. Discussion

The retrospective analysis included 50 patients with recurrent or metastatic advanced EC who received sintilimab-based regimens in a real-world clinical context. In all patients, ORR and DCR were 60% and 92%, respectively, median PFS was 11.3 months, and median OS was not reached.

Several recent clinical trials have demonstrated the efficacy of PD-1 inhibitors plus chemotherapy in the first-line treatment of advanced EC, so the treatment regimens for advanced EC are rapidly changing. In the KEYNOTE-590 trial, first-line pembrolizumab plus chemotherapy improved ORR and median OS compared with placebo plus chemotherapy (45% vs. 29.3%, 12.4 months vs. 9.8 months) [23]. Also, in the CKECKMATE-648 trial, nivolumab plus chemotherapy improved ORR and median OS compared with placebo plus chemotherapy (47% vs. 27%, 13.2 months vs. 10.7 months) [24]. The ESCORT-1st trial demonstrated that camrelizumab plus chemotherapy increased ORR and median OS compared with placebo plus chemotherapy (72.1% vs. 62.1%, 15.3 months vs. 12 months) [25]. In the ORIENT-15 trial, 659 patients were randomly divided into sintilimab combined with chemotherapy and placebo combined with chemotherapy. The ORR and median OS of the sintilimab group were better than those of the placebo group (66.1% vs. 45.5%, 16.7 months vs. 12.5 months) [26]. The ORR of all populations in this study was 60%, which was lower than 66.1% of ORIENT-15. The possible reason was that 28% of the patients received second- or third-line therapy in our study. Among the 36 patients who received first-line treatment, the ORR was 66.7% (24/36), similar to ORIENT-15 results.

Several preclinical studies have demonstrated that radiotherapy combined with immunotherapy has three major benefits: (1) radiotherapy can regulate the tumor microenvironment and increase the infiltration of cytotoxic T lymphocytes, thereby enhancing the effect of tumor regression and achieving better local control; (2) produce effector and memory immune cells to maintain antitumor immunity, thereby avoiding tumor recurrence and prolonging local control time; and (3) induce “distant effect” and reduce the risk of distant metastasis [27–29]. In a phase 2 trial in Korea, 28 patients with stage Ib-III ESCC received chemoradiotherapy along with pembrolizumab, followed by surgery and postoperative pembrolizumab maintenance therapy. The pathological complete response (pCR) rate of the primary tumor was 46.1%, whereas the 1-year survival rate was 82.1% [30]. The PALACE-1 clinical trial observed the safety and efficacy of pembrolizumab combined with chemoradiotherapy in 20 patients with resectable ESCC. The results showed that the regimen was safe and feasible, and the pCR rate was 55.6% [31]. Zhang et al. found that the ORR of camrelizumab plus radiotherapy for locally advanced EC was 74%, the median PFS was 11.7 months, and the median OS was 16.7 months [32]. A phase 1B trial showed that the ORR of concurrent chemoradiotherapy combined with camrelizumab in the treatment of locally advanced EC was 65%, with OS and PFS of 8.2-28.5 months and 4.0-28.5 months, respectively [33]. Other clinical trials of chemoradiotherapy combined with immunotherapy for EC include KEYNOTE975, ESCORT-CRT, and RATIONAL-311. We look forward to the announcement of the above research results. There is no published article on immunotherapy combined with radiotherapy for the treatment of advanced EC, but in clinical practice, radiotherapy is often used for salvage or palliative treatment of locally recurrent or metastatic advanced EC. In this study, the CR rate of immunotherapy combined with radiotherapy was 25% (6/24), which was higher than that of patients who did not undergo radiotherapy, although the median survival was not achieved.

A notable issue in this study was that patients who received immunotherapy plus radiotherapy had better OS than those who did not receive radiotherapy, but PFS was not statistically different. CHECKMATE-648 also found the same situation, the mOS of nivolumab in combination with chemotherapy was superior to that of chemotherapy (13.2 months vs. 10.7 months, HR = 0.74 (0.58–0.96)), but there was no statistical difference in mPFS between the two groups (5.8 months vs. 5.6 months, HR = 0.81 (0.64-1.04)) [24]. One probable explanation is that it is difficult to appropriately evaluate the immunotherapy response using the previous solid tumor response evaluation standards. Different from traditional treatment, immunotherapy has the particularity of response, that is, unconventional response mode, such as delayed response, pseudoprogression, mixed remission, and hyperprogression [34]. In addition to RECIST1.1 as the primary criterion, there are also several secondary criteria. In clinical practice and trials, the evaluation criteria of immunotherapy efficacy have not been unified. Additional clinical trials are still required to identify biomarkers that can predict immunotherapy efficacy. At present, a predictive model for evaluating the long-term survival of esophageal cancer has been developed, and developing a model that can predict the efficacy of immunotherapy for esophageal cancer may be a future research direction [35].

ORIENT-15 trial showed that grade 1-2 treatment-related AEs of sintilimab combined with chemotherapy were mainly anemia, decrease in white blood cell count, nausea, and vomiting. The most common grade 3-4 AEs were neutropenia, leukopenia, and anemia [26]. Treatment-related AEs in this study were similar to ORIENT-15 results, except for the incidence of pneumonia. The incidence of grades 1-2 and grades 3-4 pneumonia in this study were 34% and 10%, respectively, higher than the incidence of <1% and 3% in ORIENT-15. Li et al. [36] conducted a meta-analysis of 11 prospective clinical trials (1113 cases) of thoracic radiotherapy combined with immunotherapy for NSCLC and found that the incidence of pneumonia of all grades was 23%, and that in grades 3-5 was 3.8%, which validated the safety of radioimmunotherapy. However, it should be noted that the incidence of radiation-immune-associated pneumonia in real-world studies is higher than in clinical studies. Thomas et al. [37] retrospectively analyzed 123 patients with locally advanced NCSCL who received consolidation therapy with durvalumab in the same treatment pattern as in the PACIFIC study. The incidence of asymptomatic pneumonia was 39.8%, and the incidence of grades 3-4 symptomatic pneumonia was 13.1%, higher than the incidence of pneumonia in the PACIFIC study. Therefore, in the real world, it is necessary to strictly screen the radioimmunotherapy population, strictly observe adverse reactions, and timely management.

However, some shortcomings should be noted when interpreting our results, including retrospective study design, relatively short observation period, and small number of patients. A well-designed prospective trial with large sample size should be conducted based on these preliminary findings.

In summary, sintilimab is widely used in real-world practice because of its availability. We demonstrated that the application of sintilimab in advanced EC patients has a certain survival benefit, and adverse events can be tolerated, and combined with local radiotherapy can improve CR rate and overall survival time.

## Figures and Tables

**Figure 1:** Tumor response in 50 patients. (a) Best changes from baseline in measurable target lesions. (b) Longitudinal changes in measurable target lesions. CR: complete response; PR: partial response; SD: stable disease; PD: progressive disease.

**Figure 2:** Survival analysis in 50 patients. (a) Kaplan–Meier curves of progression free survival (PFS) for the entire study cohort. (b) Kaplan–Meier curves of overall survival (OS) for the entire study cohort. (c) Kaplan–Meier curves of PFS for the patients with or without radiotherapy. (d) Kaplan–Meier curves of OS for the patients with or without radiotherapy.

**Figure 3:** Comparison of imaging findings in a patient who was diagnosed with advanced esophageal cancer with lung and liver metastases at the first visit and received sintilimab-based regimens. (a, c, e–g) Imaging findings before treatment with 2 cycles of sintilimab plus albumin-bound paclitaxel, nedaplatin, and palliative radiotherapy for esophageal tumors (5 March 2021). (b, d, h–j) Positron emission tomography-CT showed that all lesions and tumor metabolic activity disappeared after treatment (27 May 2021).

**Table 1:** Patient demographics and clinical backgrounds.

Category or variable	No. (%) or value
No. of patients	50
Gender	
Male	34 (68.0)
Female	16 (32.0)
Age (years)	
Median	69
Range	41–85
Primary esophageal cancer	
Cervical and upper thoracic	8 (16.0)
Middle thoracic	34 (68.0)
Lower thoracic	8 (16.0)
Histology	
Squamous cell carcinoma	48 (96.0)
Adenocarcinoma	2 (4.0)
Differentiation	
Well	6 (12.0)
Moderate	23 (46.0)
Poor	2 (4.0)
Unknown	19 (38.0)
Metastasis	
Yes	36 (72.0)
No	14 (28.0)
Metastatic site	
Bone	3 (6.0)
Liver	7 (14.0)
Lung	8 (16.0)
Nonregional lymph node	21 (42.0)
Other	3 (6.0)
Esophagectomy	
Yes	28 (56.0)
No	22(44.0)
Prior radiotherapy	
Yes	5 (10.0)
No	45 (90.0)
ECOG performance status	
0	21 (42.0)
1	29 (58.0)

**Table 2:** Treatment patterns of sintilimab.

Category or variable	No. (%) or value
No. of patients	50
Treatment line	
1st line	36 (72.0)
2nd line	9 (18.0)
3rd line	5 (10.0)
Systemic treatment	
Sintilimab alone	1 (2.0)
Sintilimab plus chemotherapy	44 (88.0)
Paclitaxel	2 (4.0)
Paclitaxel plus platinum	3 (6.0)
Albumin-bound paclitaxel	3 (6.0)
Albumin-bound paclitaxel plus platinum	24 (48.0)
S-1 (tegafur-gimeracil-oteracil potassium)	4 (8.0)
S-1 plus platinum	4 (8.0)
Oxaliplatin	1 (2.0)
Irinotecan	3 (6.0)
Sintilimab plus antiangiogenic therapy	5 (10.0)
Anlotinib	3 (6.0)
Apatinib	2 (4.0)
Combination of radiotherapy	
Yes	24 (48.0)
No	26 (52.0)
Cycle of sintilimab (times)	
Median	5
Range	2–27
Duration of sintilimab (days)	
Median	119
Range	42–636

**Table 3:** Efficacy of sintilimab for recurrent or metastatic advanced esophageal cancer.

Category or variable	With radiotherapy	Without radiotherapy	*P* value	All patients
	*n* = 24	*n* = 26		*n* = 50
CR	6 (25.0)	1 (3.8)	0.031	7 (14.0)
PR	8 (33.3)	15 (57.7)		23 (46.0)
SD	8 (33.3)	8 (30.8)		16 (32.0)
PD	2 (8.3)	2 (7.7)		4 (8.0)
ORR (%)	58.3 (14/24)	61.5 (16/26)	0.817	60 (30/50)
DCR (%)	91.7 (22/24)	92.3 (24/26)	0.933	92 (46/50)

Data are number (%) or value. CR: complete response; PR: partial response; SD: stable disease; PD: progressive disease; ORR: objective response rate; DCR: disease control rate.

**Table 4:** Adverse events related to treatment based on CTCAE 5.0.

Adverse events	Grades 1-2	Grade 3	Grade 4
Anemia	35 (70.0)	2 (4.0)	0
Decrease in white blood cell count	31 (62.0)	1 (2.0)	0
Nausea/vomiting	26 (52.0)	2 (4.0)	0
Hypoproteinemia	21 (42.0)	0	0
Decrease in neutrophil count	18 (36.0)	7 (14.0)	0
Pneumonia	17 (34.0)	4 (8.0)	1 (2.0)
Decrease in platelet count	14 (28.0)	1 (2.0)	1 (2.0)
Increase in bilirubin	9 (18.0)	0	0
Increase in alanine aminotransferase	4 (8.0)	3 (6.0)	0
Rash	4 (8.0)	1 (2.0)	0
Increase in creatinine	3 (6.0)	1 (2.0)	0
Increase in aspartate aminotransferase	3 (6.0)	2 (4.0)	0

Data are number (%).

## Data Availability

All the underlying data supporting the results of our study are in the manuscript.
